# Digital imaging of colon tissue: method for evaluation of inflammation severity by spatial frequency features of the histological images

**DOI:** 10.1186/s13000-015-0389-7

**Published:** 2015-09-15

**Authors:** Robertas Petrolis, Rima Ramonaitė, Dainius Jančiauskas, Juozas Kupčinskas, Rokas Pečiulis, Limas Kupčinskas, Algimantas Kriščiukaitis

**Affiliations:** Neuroscience Institute, Lithuanian University of Health Sciences, Eiveniu str. 2, LT 50009 Kaunas, Lithuania; Institute for Digestive Research, Lithuanian University of Health Sciences, Kaunas, LT 44307 Lithuania; Clinic of Pathology, Lithuanian University of Health Sciences, Kaunas, LT 50009 Lithuania; Department of Gastroenterology, Lithuanian University of Health Sciences, Kaunas, LT 50161 Lithuania; Lithuanian University of Health Sciences, Kaunas, LT 50009 Lithuania; Department of Physics, Mathematics and Biophysics, Lithuanian University of Health Sciences, Kaunas, LT 50009 Lithuania

## Abstract

**Background:**

The efficacy of histological analysis of colon sections used for evaluation of inflammation severity can be improved by means of digital imaging giving quantitative estimates of main diagnostic features. The aim of this study was to reveal most valuable diagnostic features reflecting inflammation severity in colon and elaborate the evaluation method for computer-aided diagnostics.

**Methods:**

Tissue specimens from 24 BALB/c mice and 15 patients were included in the study. Chronic and acute colon inflammation in mice was induced by oral administration of dextran sulphate sodium (DSS) solution, while mice in the control group did not get DSS. Human samples of inflamed colon tissue were obtained from patients with ulcerative colitis (*n* = 6). Non-inflamed colon tissue of control subjects (*n* = 9) was obtained from patients with irritable bowel syndrome or functional obstipation. Analysis of morphological changes in mice and human colon mucosa was performed using 4-μm haematoxylin-eosin (HE) sections. The features reflecting morphological changes in the images of colon mucosa were calculated by convolution of Gabor filter bank and array of pixel values. All features were generalized by calculating mean, histogram skewness and entropy of every image response. Principal component analysis was used to construct optimal representation of morphological changes.

**Results:**

First principal component (PC1) was representing the major part of features variation (97 % in mice and 71 % in human specimens) and was selected as a measure of inflammation severity. Validation of new measure was performed by means of custom-made software realizing double blind comparison of differences in PC1 with expert’s opinion about inflammation severity presented in two compared pictures. Overall accuracy of 80 % for mice and 67 % for human was reached.

**Conclusion:**

Principal component analysis of spatial frequency features of histological images may provide continuous scale estimation of inflammation severity of colon tissue.

## Background

Ulcerative colitis (UC) is a chronic relapsing-remitting inflammatory disorder affecting intestinal mucosa. The pathogenic mechanisms of UC are complex and involve interaction between genetic, host immune system and environmental factors [1–3]. The diagnosis of UC is determined by standard clinical, endoscopic, radiological, and histological criteria [4]. Histological analysis is an important component in diagnosis, classification, and evaluation of treatment effectiveness of UC [5]. Several scoring schemes for images of haematoxylin–eosin (HE) stained sections are currently used in inflammatory bowel diseases and classification of colon inflammation activity. Some histological scoring schemes are designed particularly for UC cases [6–10]. Analysis of microscopy images and histological scoring is not only time consuming, but the results are often susceptible to inconsistency due to human factor [11, 12]. Development of digital microscopic imaging technology and image processing techniques [13] inspired research towards translational computational systems that can detect, analyze, classify, and quantify tissue sections. Usage of digital imaging systems could make histological image assessment less time consuming, but also could improve diagnostic quality due to objective estimation of image features.

Histological features of chronic active UC listed in the guidelines for visual inspection and evaluation of histologic images include crypt distortion, crypt branching, and lymphoplasmacytic infiltration deep into the crypts [14]. It is possible to elaborate quantitative estimates of these and similar features based on mathematical transforms used for pattern evaluation in the images from various technical areas, e.g. defect detection in textile [15] or medical diagnostics, e.g. detection of early stage of cancer in human cervical tissues [16]. The approach mentioned above is based on estimation of spatial frequency parameters of the images and provides quantitative estimates of periodic and/or random structures. Majority of known diagnostic features of UC could also be considered as estimates of periodic and/or random structures. Therefore, methods aimed at evaluation of spatial frequency parameters could provide promising results.

The aim of this study was to develop a method for automated evaluation of inflammation severity based on evaluation of spatial frequency features in histological images of inflamed mice and human colon tissue.

## Methods

### Animals and experimental colitis model

BALB/c mice used in this study come from our previous research that aimed to evaluate the role of NADPH oxidase in pathogenesis of colon inflammation [17]. Acute and chronic colon inflammation in the animals was induced by oral administration of 3.5 % dextran sulphate sodium (DSS, TdB Consultancy, Uppsala, Sweden). Detailed methods of experimental colitis induction in mice and clinical data analysis have been published in R. Ramonaite et al. paper [17] and our current study included only histological samples of the colon. Lithuanian Animal Ethics Committee approved the design of experiments (Protocol no. 0201).

### Histological specimen imaging

Images were taken by means of OLYMPUS IX71 light microscope (×20 magnification) equipped with Q IMAGING EXI aqua camera at 1392 × 1040 pixels resolution (0.6 μm/pixel).

### Assessment of the histological score in mice

Colonic segments were washed with the Mg^+2^ or Ca^+2^ free phosphate-buffered solution (PBS) and immediately fixed by the neutral 10 % formalin for 4 h at room temperature for paraffin embedding. Serial 4-μm sections were cut for each tract and stained with HE. The experts approved the image resolution for further analysis, confirming that all the tissue levels and structures are not distorted and clearly visible. Histological examination was performed using analysis method according to M. Hausmann et al. [18].

### Patients

Fifteen subjects participated in the study: 6 patients with UC (medium age (year ± SD) = 42 ± 20.85, men *n* = 4, women *n* = 2) and 9 control subjects (medium age (year ± SD) = 64.44 ± 15.73, men *n* = 5, women *n* = 4). UC patients and control subjects were recruited in the Department of Gastroenterology, Hospital of Lithuanian University of Health Sciences during the years 2011–2014. The diagnosis of UC was based on standard clinical, endoscopic, radiological, and histological criteria [19–21]. Patients with mild to severe disease activity were included in the study (Mayo UC Endoscopic Score 1 to 3). The control group consisted of patients with irritable bowel disease or functional constipation and routine colonoscopy was performed as a part of their planned examination workup. Individuals were included in the control group if they had a no endoscopic signs of inflammation during colonoscopy. Kaunas Regional Biomedical Research Ethics Committee approved inclusion of patients within the study (Protocol No. BE-2-10).

### Assessment of histological score in humans

The colon biopsies were obtained from inflamed (UC patients) and non-inflamed mucosa (control subjects) during endoscopy. Biopsies were washed with the PBS and immediately fixed by the neutral 10 % formalin for 4 h at room temperature for paraffin embedding. Serial 4-μm sections were cut for each tract stained with HE and examined using Riley scoring technique [8].

### Statistical analysis

All clinical and histological data were analyzed using SPSS version 16.0 software (SPSS Inc., Chicago, IL). Statistical analyses were performed using one-way ANOVA according to *Ramonaite* et al. [3, 17].

### Image preprocessing

Image processing algorithms were realized as programs in MATLAB computation environment and ran on personal computer with an Intel® Core™ 2 Duo, 3.06 GHz processor and 2GB of RAM.

Normalization of illumination intensity in images was realized by means of image histogram alignment using algorithm similar to Petrolis et al. [22]. All images contained empty white areas with no cells, the pixel values of which were forming a peak on the right side of the image histogram used as the reference. Image illumination adjustment was made adding certain bias to pixel values. The bias value was determined by maximizing correlation between histogram peaks representing white areas in analyzed pictures and ones in reference image. All analyzed pictures were preprocessed with the same procedure.

Automatic image features formation was performed on 512 × 512 pixel mice and human colon image cutouts (samples) selected by the experts, representing as much as possible homogeneous and typical tissue pattern without any gaps. Fifty such samples were representing acute inflammation, 50 chronic inflammation and 50 healthy controls for mice specimen cutouts. One-hundred-fifty-six samples were representing UC and 96 came from controls of human biopsy images.

Examples of typical images representing whole range of tissue patterns form healthy controls to acute inflammation and their cutouts are presented in top and middle rows of Fig. 1.

**Fig. 1:** Examples of typical analyzed images representing whole range of tissue patterns: healthy control (**a**–mice; **f**–human) on the *left*; chronic inflammation (**b**–mice; **g**–human) in the *middle* and acute inflammation (**c**–mice; **h**–human) in the *right*. Examples of image cutouts used for analysis are below the whole sample images (from *A1* to *H2*). Graph (**e**) and image of typical Gabor function (**d**) in the *middle row*

### Algorithm for feature extraction

Main diagnostic features in histologic images characterizing UC include crypt distortion, branching, and appearance of lymphoplasmacytic infiltrate deep in the crypts [23]. In digital image representation crypts are elliptic white spots varying about 180–350 pixels long and 50–130 pixels wide, both for human and mice specimens. Appearance of eosinophils, which also might be present during inflammation, is expressed as appearance of rounded spots of 7–25 pixels in diameter for all test samples. Therefore, development of inflammatory process could be described by appearance or disappearance of certain contrasted spots of some dimensions, changes of their density and even some specific changes in tissue pattern structure. We used Gabor filters for detection and evaluation of such morphological changes. The procedure performs convolution of analyzed image with function constructed of a cosine wave modulated by two-dimensional Gaussian function [24]:

1 $$ {g}_{\uplambda, \uptheta, \upvarphi, \upsigma, \upgamma}\left(x,y\right)= \exp \left(-\frac{x{\prime}^2+{\upgamma}^2y{\prime}^2}{2{\upsigma}^2}\right) cos\left(2\uppi \frac{x^{\prime }}{\uplambda}+\upvarphi \right), $$

where *x* ′ = *x* cos θ + *y* sin θ, and *y* ′ = − *x* sin θ + *y* cos θ.

*θ* in the equations is the orientation of the Gabor function in degrees; *λ* represents the wavelength of the cosine factor; *φ* is the phase offset in degrees; *γ* is the spatial aspect ratio of elliptic Gabor function and σ is the standard deviation of the Gaussian kernel. We can construct Gabor functions similar in shape to the sought objects in the images or patterns expecting maximal Gabor filter response when applied to corresponding place in the image. That for we need to define following Gabor functions parameters: spatial frequency of the cosine factor *f* = *1*/ *λ* and half-response spatial frequency bandwidth *b* (in octaves) of a Gabor filter. The last is related to the ratio σ / λ as follows:

2 $$ b={ \log}_2\frac{\frac{\upsigma}{\uplambda}\uppi +\frac{\sqrt{ \ln 2}}{2}}{\frac{\upsigma}{\uplambda}\uppi -\frac{\sqrt{ \ln 2}}{2}}, $$

where ratio σ / λ is expressed as:

3 $$ \frac{\upsigma}{\uplambda}=\frac{1}{\uppi}\frac{\sqrt{ \ln 2}}{2}\frac{2^b+1}{2^b-1}. $$

According to recommendations given in [24] we used following parameters to construct Gabor filter bank:

*φ*: 0
*θ*: 0°, 30°, 60°, 90°, 120°, 150°
*γ*: 0.5, 2, 4
*λ*: 20, 30, 40
*b*: 5 octaves, 10 octaves, 15 octaves, 20 octaves.

The example of Gabor function is presented on the bottom of Fig. 1. It is easy to recognize similarity between the shape of Gabor function and certain objects of interest in analyzed images, e.g. crypts, neutrophils, abnormalities of the muscularis mucosae, increase of the cells in transmucosal lamina propria, etc.

### Assessment of inflammation in digital images cutouts

Constructed filter bank consisted of 216 filters in total (6 orientations; 3 spatial aspect ratios; 3 wave lengths; 4 frequency bandwidths). Application of each filter to ordinary 512 × 512 pixels sample image produced 512 × 512 arrays of responses corresponding to particular spatial aspect ratios, wavelengths and frequency bandwidths for each of 6 orientations. Only the maximal values of responses in regard to orientations were taken for further analysis compensating initial arbitrary orientation of tissue structure in the analyzed image. After this operation we have 36 arrays of 512 × 512 filter responses representing each sample image. We generalized these features calculating mean, histogram skewness and entropy of every responses array, finally getting array of 108 features (36 triplets) representing each analyzed sample image. Mean was calculated:

4 $$ mean=\frac{1}{mn}\sum_{i=1}^m\sum_{j=1}^n{x}_{ij} $$

where x_ij_ is pixel value of *i*^th^ row and *j*^th^ column of analyzed image cutout; m–number of rows and n–number of columns of analyzed image cutout.

Histogram skewness was calculated:

5 $$ skewness=\frac{\frac{1}{mn}\sum_{i=1}^m\sum_{j=1}^n{\left({x}_{ij}-\overline{x}\right)}^3}{s^3} $$

where x_ij_ is pixel value of *i*^th^ row and *j*^th^ column of analyzed image cutout; m–row number and n–column number of analyzed image cutout; x̅–mean of pixel values of analyzed image cutout.

Entropy was calculated:

6 $$ entropy=-{\displaystyle \sum_{i=1}^n\left({p}_i\cdot { \log}_2\left({p}_i\right)\right)}, $$

where p_i_ is normalized *i*^th^ bin value of histogram of analyzed image cutout.

Pooling all data representing analyzed images arrays which contained data representing several cutouts of images taken from several histological pictures of each investigative. It means, one can expect the data array to be not homogeneous and independent, but rather a mixture of several clusters. Testing null-hypothesis about equality of distributions of parameter values in all hierarchal levels (between histological pictures and between investigatives) proved homogeneity of these arrays (Kruskal-Wallis test, *p* > 0.1). Array of features representing all sample images formed 150 × 108 matrix (108 features form 150 images) for mice and 252 × 108 (108 features from 252 images) matrix for human specimens:

7 $$ X=\left[\begin{array}{cccc}\hfill {x}_{1,1}\hfill & \hfill {x}_{1,2}\hfill & \hfill \cdots \hfill & \hfill {x}_{1,m}\hfill \\ {}\hfill {x}_{2,1}\hfill & \hfill {x}_{2,2}\hfill & \hfill \cdots \hfill & \hfill {x}_{2,m}\hfill \\ {}\hfill \cdots \hfill & \hfill \cdots \hfill & \hfill {x}_{i,j}\hfill & \hfill {x}_{i,m}\hfill \\ {}\hfill {x}_{n,1}\hfill & \hfill {x}_{n,1}\hfill & \hfill \cdots \hfill & \hfill {x}_{n,m}\hfill \end{array}\right], $$

where x_i,j_ is the *j*^th^ feature of *i*th image cutout. Principal component analysis (PCA) transforms original feature data set X into new space of variables maximizing variation and concentrating correlated original variables [25]. Our training sets of images were constructed so that variation in feature values in regard to inflammation intensity takes the biggest part in it. Then we expect that first or at least one of the first computed new variables (principal components) will give optimal quantitative estimate of inflammation. Spatial correlation R of original representation of all images feature data set X can be estimated as:

8 $$ {R}_X=\frac{1}{n\cdot m}X\cdot {X}^T $$

The eigenvector equation for *R*_*X*_ [25], representing variation of original feature data set **X**, is:

9 $$ {R}_X\cdot \uppsi =\uppsi \cdot \varLambda $$

where Λ denotes the eigenvalue matrix with the eigenvalues sorted in descending order, and Ψ is the corresponding eigenvector matrix. The matrix Ψ defines an orthonormal transform, which is applied to the original data X and principle component matrix Y is computed:

10 $$ Y={\uppsi}^T\cdot X. $$

The first principal component (PC1) appears in first row of matrix Y and we will use it as quantitative estimate of inflammation.

To validate this new constructed variable, estimated for human and mice specimens separately, experts participated in double blind experiment realized by means of special software created in JAWA programing language. The program shows two randomly selected images for the expert, asking him to select the one corresponding to more severe inflammation. The choice of the expert is stored together with values of PC1 corresponding to shown images. Screenshot of the program window is shown on Fig. 2.

**Fig. 2:** Screenshot of developed program for double blinded validation of computed inflammation severity measure by comparing it to expert’s opinion

## Results

### Histological assessment of colon inflammation in mice

Oral administration of 3.5 % DSS solution for 7 days induced severe acute colitis in mice with significant morphological alterations in the colon mucosa. We determined inflammatory cell infiltration of L. submucosa (3.8 ± 0.46) and major epithelium damage with loss of crypts in large areas (3.9 ± 0.38) in mice colon tissue with acute colitis. Administration of 3.5 % DSS for 44 days induced less severe damage of colon tissues, however, inflammatory cell infiltration of L. muscularis mucosae (2.3 ± 0.31) and loss of goblet cells in large areas (2.8 ± 0.16) were observed. Control mice possessed no histological alterations in the colon tissues (Table 1).

**Table 1:** Histological characteristics of BALB/c mice colon tissue

Group	*n*	Epithelium damage	Inflammatory cells infiltration
Control	10		
Means		0.2 ± 0.25	0.2 ± 0.18
Min/max ranges		0 to 1	0 to 1
Acute colitis	7		
Means		3.9 ± 0.38 ^a^	3.8 ± 0.46 ^a^
Min/max ranges		2 to 4	2 to 4
Chronic colitis	7		
Means		2.8 ± 0.16 ^a^ ^b^	2.3 ± 0.31 ^a^ ^b^
Min/max ranges		1 to 3	1 to 3

Analysis of histological parameters was performed as described in Methods. ^a^Statistically significant difference between control and dextran sulphate sodium (DSS)-induced colitis groups (*P* <0.05). ^b^ Statistically significant difference between acute DSS-induced colitis and chronic DSS-induced colitis groups (*P* <0.05)

### Histological assessment of colon inflammation in humans

We determined crypt abscesses, (1.50 ± 0.55) epithelial integrity (2.17 ± 0.75) and crypt architectural (2.00 ± 0.63) irregularities together with inflammatory cell infiltration (acute inflammatory cell infiltrate was assessed 1.83 ± 0.75; chronic inflammatory cell infiltrate–2.33 ± 0.82) and mucin depletion (2.33 ± 0.82) in colon mucosa of patients with UC. Control subjects had no or minor histological alterations in the colon tissues. Analysis of histological parameters showed statistically significant differences between control and UC groups (Table 2).

**Table 2:** Histological characteristics of human colon tissue

	*n*	Acute inflammatory cell infiltrate	Chronic inflammatory cell infiltrate	Crypt abscesses	Mucin depletion	Surface epithelial integrity	Crypt architectural irregularities
UC	6						
Means		1.83 ± 0.75	2.33 ± 0.82	1.50 ± 0.55	2.33 ± 0.82	2.17 ± 0.75	2.00 ± 0.63
Min/max ranges		1 to 3	1 to 3	1 to 2	1 to 3	1 to 3	1 to 3
Control	9						
Means		0.25 ± 0.46^#^	0.38 ± 0.52^#^	0.00 ± 0.00^#^	0.13 ± 0.35^#^	0.13 ± 0.35^#^	0.00 ± 0.00^#^
Min/max ranges		0 to 1	0 to 1	0	0 to 1	0 to 1	0

Analysis of histological parameters was performed as described in Methods. ^#^ Statistically significant difference between control and ulcerative colitis (UC) groups (*P* <0.05)

### Assessment of PC1 ordered digital images cutouts for inflammation

Principal Component Analysis transformed characterization of all sample images from 108 features space, into optimal variables (‘Principal Components’) space. PC1 was representing the major part (97 % in mice and 71 % in human specimens) of total variation. Exact percentage of contribution of each principal component is shown in Fig. 3.

**Fig. 3:** Contribution percentage of total feature variation of the first ten principal components

We normalized obtained values of PC1 corresponding to all images into [0, 1] range and considered it as the inflammation severity measure. Maximal value “1” was corresponding most severe inflammation and “0”–no inflammation (control). Ordered values of PC1 are presented in Fig. 4 together with several sample images, corresponding to certain values of PC1. Whole set of sample images ordered according to their corresponding values of PC1 are shown on Fig. 5.

**Fig. 4:** Computed first principal component (PC1) values with analysed images, corresponding to certain values of it

**Fig. 5:** Set of analyzed images ordered according to their computed first principal component (PC1) values. Composed pictures are starting with healthy control cutouts from mice and human specimens at *top left* images and ends with most severe inflammation at *bottom right* images

Three histology experts participated in double blind validation of proposed inflammation severity measure using custom made software. The software was showing randomly selected images corresponding to different values of PC1 and registered opinion of the expert which of them was corresponding to more severe inflammation. Expert’s opinion was matching with decision according PC1 values in 79.9 % of 3402 mice image pairs of specimen and in 67 % of 5796 human image pairs of specimen covering whole range of PC1 values. Absolute matching was in cases when difference in PC1 values was maximal. Dependency of ratio of expert’s opinion mismatching with difference in PC1 values is shown in Fig. 6. The highest yet acceptable ratio indicates resolution of our method.

**Fig. 6:** Mismatch ratio between expert’s decision and first principal component (PC1) values

Proposed measure of inflammation severity–first Principal Component, is constructed by convolution of first eigenvector with initial set of features (see formula (7)). Therefore, values of its elements reflect contribution of particular features for constructed optimal representation. Values of first eigenvector corresponding to each particular feature (mean, histogram skewness or entropy at certain spatial frequency or spatial aspect ratio) are shown in Fig. 7. Highest values were found at positions corresponding to features representing objects similar to eosinophils (rounded spots about 7–25 pixels in diameter). Interestingly, Gabor functions corresponding to objects similar to crypts (elliptic spots varying about 180–350 pixels long and 50–130 pixels wide) were not expressed as important.

**Fig. 7:** Values of first eigenvector corresponding to each particular feature: mean (marked with *diamonds*); analyzed image histogram skewness (marked with *circles*) or analyzed image entropy (marked with *asterices*) at certain spatial frequency and aspect ratio

## Discussion

Several studies have shown that image processing and analysis systems may be successfully used for diagnosis and classification of various diseases, such as neuroblastoma, melanoma, lung, prostate, and breast cancer. However, these computerized analysis systems are based mainly on color-space derived features of histological images and indicate only areas with positive or negative diagnostic result [26–30] ignoring morphological properties of specimen. In this study, we presented a new method for automated evaluation of inflammation severity based on spatial frequency features extracted from histological images of mice and human colon tissue. Developed technique computed quantitative estimate of inflammation severity and constructed a continuous scale estimate of it.

Currently published guidelines for visual evaluation of histological preparations of colon tissue describe expert scoring schemes enabling to classify severity of inflammation into several grades [8, 10, 31]. Our idea of elaboration of possibly continuous scale measure for inflammation severity was based on presumption that even specimens from the same investigative could represent certain variety of inflammation severity. The same principle concerns image cutouts from the same histological preparation. This presumption was supported by experts pathologists, who observed certain variety of visually evaluated features within cases classified into one or another class according to currently used scoring techniques. So we decided to pool all data, construct continuous scale measure and test it by simplified question to the experts during double blind experiment showing them two randomly selected images and asking: “just use your experience and select image representing more severe inflammation”. That experiment confirmed suitability of our measure. Pooling all data representing analyzed images arrays contained data representing several cutouts of images taken from several histological pictures of each investigative. It means, one can expect the data array to be not homogeneous and independent, but rather a mixture of several clusters. Therefore we tested and retained null-hypothesis about equality of distributions of used data from these several clusters (Kruskal-Wallis test).

At the moment we do not have any “golden standard” method for verification of our results, so determination of resolution achieved by our method could be based on maximal yet acceptable value of discordance between expert’s opinion in double blind test and our principal component analysis based estimate. The estimation of maximal yet acceptable value of mismatch ratio could be detected by evaluation of concordance between opinions of different experts on the same image pairs. However, this requires recruitment of many experts into the experiment and should be an interesting task of further research in this field. Detailed analysis of eigenvector values reveals diagnostic value of particular features and could be used for optimization of initial feature set for processing. Particular disease is related with unique tissue structure and changes of it in progress of disease. So, using our methodology we can elaborate disease progress measures for other diseases as well.

Currently, clinical, endoscopic, radiological, histological criteria and molecular markers are used to evaluate inflammation severity of colon in UC patients. Estimates obtained from standard clinically approved features could be also used for verification of our method. However, registration of such estimates “in vivo” is technically difficult and such combined experiments remain an interesting topic for future research. We show that complex evaluation of colon inflammation severity using computer-aided analysis could reveal new alternatives for evaluation of the degree of inflammation severity with higher precision and may provide new diagnostic possibilities.

## Conclusions

Quantitative evaluation of inflammatory changes in histological preparations of colon tissues is feasible by estimation of spatial frequency parameters of histological images. Principal component analysis of the spatial frequency features improves efficacy of estimation of inflammation severity of colon tissue. The method may have potential clinical applications in patients with colon inflammation.

## Abbreviations

PCA: Principal component analysis
PC1: First principal component obtained by principal component analysis of image features
UC: Ulcerative colitis
DSS: Dextran sulphate sodium
HE: Haematoxylin-eosin
NADPH: Nicotinamide adenine dinucleotide phosphate
PBS: Free phosphate-buffered solution

## References

[1] Cooney R, Jewell D (2009). The genetic basis of inflammatory bowel disease. Dig Dis.

[2] Davies JM, Abreu MT (2015). The innate immune system and inflammatory bowel disease. Scand J Gastroenterol.

[3] Ramonaite R, Skieceviciene J, Kiudelis G, Jonaitis L, Tamelis A, Cizas P (2013). Influence of NADPH oxidase on inflammatory response in primary intestinal epithelial cells in patients with ulcerative colitis. BMC Gastroenterol.

[4] Bressenot A, Geboes K, Vignaud JM, Guéant JL, Peyrin-Biroulet L (2013). Microscopic features for initial diagnosis and disease activity evaluation in inflammatory bowel disease. Inflamm Bowel Dis.

[5] Geboes K, Dalle I (2002). Influence of treatment on morphological features of mucosal inflammation. Gut.

[6] Danielsson A, Hellers G, Lyrenas A, Löfberg R, Nilsson Å, Olsson O (1987). A controlled randomized trial of budesonide versus prednisolone retention enemas in active distal ulcerative colitis. Scand J Gastroenterol.

[7] Riley SA, Mani V, Goodman MJ, Herd ME, Dutt S, Turnberg LA (1988). Comparison of delayed release 5 aminosalicylic acid (mesalazine) and sulphasalazine in the treatment of mild to moderate ulcerative colitis relapse. Gut.

[8] Riley SA, Mani V, Goodman MJ, Dutt S, Herd ME (1991). Microscopic activity in ulcerative colitis: what does it mean?. Gut.

[9] Gomes P, Du Boulay C, Smith CL, Holdstock G (1986). Relationship between disease activity and colonoscopic findings in patients with colonic inflammatory bowel disease. Gut.

[10] Bressenot A, Salleron J, Bastien C, Danese S, Boulagnon-Rombi C, Peyrin-Biroulet L (2015). Comparing histological activity indexes in UC. Gut.

[11] Conway C, Dobson L, O’Grady A, Kay E, Costello S, O’Shea D (2008). Virtual microscopy as an enabler of automated/quantitative assessment of protein expression in TMAs. Histochem Cell Biol.

[12] Ong CW, Kim LG, Kong HH, Low LY, Wang TT, Supriya S (2010). Computer-assisted pathological immunohistochemistry scoring is more time-effective than conventional scoring, but provides no analytical advantage. Histopathology.

[13] Onder D, Sarioglu S, Karacali B (2014). Automated labeling of cancer textures in larynx histopathology slides using quasi-supervised learning. Anal Quant Cytopathol Histpathol.

[14] Moussata D, Boschetti G, Chauvenet M, Stroeymeyt K, Nancey S, Berger F (2015). Endoscopic and histologic characteristics of serrated lesions. World J Gastroenterol.

[15] Kumar A, Pang GK-H (2002). Defect detection in textured materials using Gabor filters. IEEE Trans Ind Appl.

[16] Pu Y, Jagtap J, Pradhan A, Alfano R. Spatial frequency analysis for detecting early stage of cancer in human cervical tissues. Technol Cancer Res Treat. 2013; Epub ahead of print.10.7785/tcrtexpress.2013.600270PMC452746724000997

[17] Ramonaite R, Skieceviciene J, Juzenas S, Salteniene V, Kupcinskas J, Matusevicius P (2014). Protective action of NADPH oxidase inhibitors and role of NADPH oxidase in pathogenesis of colon inflammation in mice. World J Gastroenterol.

[18] Hausmann M, Obermeier F, Paper DH, Balan K, Dunger N, Menzel K (2007). In vivo treatment with the herbal phenylethanoidacteoside ameliorates intestinal inflammation in dextran sulphate sodium-induced colitis. Clin Exp Immunol.

[19] Okayasu I, Hatakeyama S, Yamada M, Ohkusa T, Inagaki Y, Nakaya R (1990). A novel method in the induction of reliable experimental acute and chronic ulcerative colitis in mice. Gastroenterology.

[20] Axelsson LG, Landström E, Goldschmidt TJ, Grönberg A, Bylund-Fellenius AC (1996). Dextran sulfate sodium (DSS) induced experimental colitis in immunodeficient mice: effects in CD4 + −cell depleted, athymic and NK-cell depleted SCID mice L.-G. Inflamm Res.

[21] Wirtz S, Neufert C, Weigmann B, Neurath MF (2007). Chemically induced mouse models of intestinal inflammation. Nat Protoc.

[22] Petrolis R, Čižas P, Borutaitė V, Kriščiukaitis A. Method of fluorescence imaging for evaluation of membrane potential in cultured neurons using transmembrane voltage sensitive dye. Biomedical Engineering 2011: Proceedings of International Conference. 2011;14:16–9.

[23] Langner C, Aust D, Ensari A, Villanacci V, Becheanu G, Miehlke S (2015). Histology of microscopic colitis-review with a practical approach for pathologists. Histopathology.

[24] Chuanzhen L, Zhang Q (2011). Improved feature for texture segmentation using Gabor filters. Communications in Computer and Information Science.

[25] Jollife IT (2002). Principal component analysis.

[26] Sieren JC, Weydert J, Bell A, De Young B, Smith AR, Thiesse J (2010). An automated segmentation approach for highlighting the histological complexity of human lung cancer. Ann Biomed Eng.

[27] Sertel O, Kong J, Shimada H, Catalyurek UV, Saltz JH, Gurcan MN (2009). Computer-aided prognosis of neuroblastoma on whole-slide images: classification of stromal development. Pattern Recognit.

[28] Orlov NV, Weeraratna AT, Hewitt SM, Coletta CE, Delaney JD, Mark Eckley D (2012). Automatic detection of melanoma progression by histological analysis of secondary sites. Cytometry A.

[29] Yu E, Monaco JP, Tomaszewski J, Shih N, Feldman M, Madabhushi A (2011). Detection of prostate cancer on histopathology using color fractals and probabilistic pairwise Markov models. Conf Proc IEEE Eng Med Biol Soc.

[30] He L, Long LR, Antani S, Thoma GR (2012). Histology image analysis for carcinoma detection and grading. Comput Methods Programs Biomed.

[31] Geboes K, Riddell R, Ost A, Jensfelt B, Persson T, Löfberg R (2000). A reproducible grading scale for histological assessment of inflammation in ulcerative colitis. Gut.

